The article "Research on multi-objective optimal scheduling considering the balance of labor workload distribution" was retracted in 2025. Reasons: compromised peer review; unreliable results or conclusions; concerns about the peer review.

# Research on multi-objective optimal scheduling considering the balance of labor workload distribution

**DOI:** 10.1371/journal.pone.0255737

**Published:** 2021-08-05

**Authors:** Zhengyu Hu, Wenrui Liu, Shengchen Ling, Kuan Fan

**Affiliations:** School of Computer and Communication Engineering, Northeastern University, Qinhuangdao, Hebei, People’s Republic of China; Ministry of Natural Resources North Sea Bureau, CHINA

## Abstract

In order to solve the problem of unbalanced workload of employees in parallel flow shop scheduling, a method of job standard balance is proposed to describe the work balance of employees. The minimum delay time of completion and the imbalance of employee work are taken as the two goals of the model. A bi-objective nonlinear integer programming model is proposed. NSGA-II-EDSP, NSGA-II-KES, and NSGA-II-QKES heuristic rule algorithms are designed to solve the problem. A number of computational experiments of different sizes are conducted, and compared with solutions generated by NSGA-II. The experimental results show the advantages of the proposed model and method, which error is reduced 14.56%, 15.16% and 15.67%.

## 1. Introduction

With the continuous development of economic globalization, manufacturing industry is gradually globalized, and manufacturing enterprises are facing unprecedented competition. In this context, in order to improve the competitiveness of enterprises, it is necessary to change from the traditional single production line to the parallel production line. Scheduling problem is a classic research problem [1–3] to improve production efficiency and reduce cost in production workshop. Parallel flow shop [4–7] refers to a production mode in which a plurality of production lines are arranged in the form of flow shop, which generally exists in cable, household appliances, automobile manufacturing, steel and other industries [8–10]. Röck [11] has proved that the flow shop scheduling problem with more than three machines is NP-complete. Therefore, parallel flow shop scheduling is also NP-complete. That is to say that there is no polynomial time exact algorithm for solving this kind of optimization problem, unless P = NP. In view of this kind of problem, a large number of scholars have proposed a variety of heuristic algorithms to solve it, such as Rule Scheduling Algorithm [12] and Evolutionary Algorithm [13], from the perspective of single objective optimization, for example, the minimum completion time or the minimum waiting time of flow shop workpieces. However, in the actual parallel flow shop scheduling process, it usually involves optimizing multiple objectives at the same time, such as machine efficiency, material waste, maximum delivery time of workpieces, etc., and each objective may be inconsistent or even conflict with each other [14]. Therefore, it is of great practical significance to introduce multi-objective optimization into parallel flow shop scheduling.

In the research of parallel flow shop scheduling, the exact algorithm’s solving time increases sharply with the increase of the problem scale, which is not suitable for solving large-scale problems and has few practical applications [15–17]. Researchers prefer approximate algorithms, including intelligent optimization algorithm, rule method and meta-heuristic algorithm [16, 18–20]. Azadeh et al. [21] take a multi-state machine flow shop manufacturing system as the background, using genetic algorithm to optimize its system has three objectives, minimizing system procurement cost, minimizing completion time and maximizing system reliability. Comparing with simulated annealing method, it proves that genetic algorithm is superior in solving such problems. Zou et al. [22] studied the two-stage three machine assembly shop scheduling problem. Zhang et al. [23] proposed an improved genetic algorithm to solve the flexible job shop scheduling problem considering the job transportation time between machines. Christoforos et al. [24] studied the non-equivalent parallel multi-machine scheduling problem aiming at minimizing the completion time. An exact solution method combining heuristic algorithm and mathematical programming is designed. Azizoglu [25] considers that the processing cost of each equipment for the same process is inconsistent, the processing cost is nonlinear with the processing time, and establishes a production scheduling model that minimizes the production cost. Jiang et al. [26] studied a flow shop scheduling problem with conveyor belt transportation and transportation time. Coorea et al. [27] considered the order priority constraint when studying the scheduling of non-equivalent parallel machines. The scheduling model is established to minimize the order completion time. Xie et al. [28] proposed a scheduling algorithm for cloud computing system based on dynamic essential path drive. Zelazny et al. [29] proposed a new parallel tabu search algorithm in the double objective optimization of minimizing the total completion time and total flow time of the replacement flow shop, and the better Pareto front solution and shorter solution time are obtained. Sheikhalishahi et al. [30] established the optimal scheduling model of worker error rate, machine utilization rate and total processing time considering worker error and preventive maintenance. Experiments show that NSGA-II has better optimization effect than multi-objective particle swarm optimization (MOPSO). Although the research on flow shop scheduling problem has been rich, the existing research focus on the optimization of time and cost objectives, ignoring the psychological imbalance caused by the difference in workload distribution, resulting in productivity reduction and turnover rate increase.

In view of this phenomenon, while considering minimizing the total delay time, this paper takes minimizing the standard deviation of the workload assigned by all employees as the goal to measure the equilibrium rate of job assignment, and designs NSGA-II-EDSP, NSGA-II-KES, and NSGA-II-QKES heuristic rule algorithms to optimize the multi-objective parallel flow shop scheduling problem based on NSGA-II algorithm, which improves the production efficiency and employee satisfaction. This paper is mainly divided into five parts. The first and second parts are introduction and mathematical model construction. The third and fourth parts are algorithm design and case solving. The last part is the summary and Prospect of the article.

## 2. Establishment of mathematical model for multi-objective flow shop scheduling

In this paper, it is assumed that a total of *p* employees are responsible for processing *n* workpieces in *j* teams and groups, and each workpiece needs to go through *m* processes in sequence. It is assumed that employees in the same process have the same operating efficiency, so each employee will share the total workload of the process. For the processes in the same team, the processing sequence of each workpiece is the same. There is a problem of Permutation Flow Shop in each shift. Any workpiece *I* has a due date *D*_*i*_, and its processing time in process *m* is *T*_*im*_, the starting processing time is *S*_*im*_, and the completion delay time of the workpiece is *T*_*i*_. The work time assigned by any employee *p* is recorded as *L*_*p*_.

According to the above assumptions and symbolic descriptions, the mathematical programming model is established as follows:

$$MinT=\sum_{i=1}^{N}T_{i}$$ (1)

$$Min\sigma =\sqrt{(\frac{1}{P}\sum_{p=1}^{P}{\left(L_{p}-\frac{1}{P}\sum_{k=1}^{P}L_{k}\right)}^{2}}$$ (2)

$$\sum_{j=1}^{J}X_{i}{}_{j}=1,i=1,\ldots ,N$$ (3)

$$S_{im}\geq S_{i,m-1},i=1,\ldots ,N,m=2,\ldots ,M$$ (4)

$$S_{i0}\geq 0,i=1,\ldots ,N$$ (5)

$$\begin{array}{l} max\left\{\begin{array}{c} \sum_{u=1}^{N}S_{u}{}_{m}*X_{uj}-\sum_{v=1}^{N}(S_{vm}-T_{vm})*X_{vj},\\ \sum_{v=1}^{N}S_{v}{}_{m}*X_{vj}-\sum_{u=1}^{N}(S_{um}-T_{um})*X_{uj} \end{array}\right\}\geq 0\\ j=1,\ldots ,J;m=1,\ldots ,M \end{array}$$ (6)

$$Tj=max\{0,S_{iM}+T_{iM}-D_{i}\}i=1,\ldots ,N$$ (7)

$$Q_{j}{}_{m}=\sum_{i=1}^{N}X_{ij}*T_{im},j=1,\ldots ,J;m=1,\ldots ,M$$ (8)

$$G_{j}{}_{m}=\sum_{p=1}^{P}Y_{pjm},j=1,\ldots ,J;m=1,\ldots ,M$$ (9)

$$Lp=\frac{\sum_{j=1}^{J}\sum_{m=1}^{M}Q_{jm}*Y_{pjm}}{\sum_{j=1}^{J}\sum_{m=1}^{M}G_{jm}*Y_{pjm}},p=1,\ldots ,P$$ (10)

$$Y_{pjm}=\{\begin{array}{l} 1,\;\mathrm{employee}\;p\;\mathrm{is}\;\mathrm{arranged}\;\mathrm{on}\;\mathrm{the}\;m\;\mathrm{workpiece}\;\mathrm{of}\;\mathrm{team}\;j\\ 0,\;others \end{array}$$ (11)

$$X_{ij}=\{\begin{array}{l} 1,\;j\mathrm{ob}\;i\;\mathrm{is}\;\mathrm{assigned}\;\mathrm{to}\;\mathrm{team}\;j\\ 0,\;others \end{array}$$ (12)

Eq (1) and Eq (2) are objective functions, and Eq (1) represents minimizing the total delay time of all workpieces, Eq (2) maximizes the equilibrium rate of assignment by minimizing the standard deviation of assignment time. Eq (3) indicates that any workpiece *i* is assigned to only one shift. Eqs (4) and (5) represent sequence constraints of processes, and for any process *m* of any shift *j*, workpiece *i* can only be processed in the next process after it has been processed in the previous process. Eq (6) is the processing sequence constraint of workpieces, and only one workpiece can be processed at the same time in any process *M* of any shift *J*, so for any two workpieces *U* and *V*, the processing start and end time has a sequence constraint. Eq (7) calculate the delay time of any workpiece *i*. In Eq (8), *Q*_*jm*_ represents the sum of the operation time allocated by the process *m* of any shift *j*. *G*_*jm*_ in Eq (9) indicates the number of employees configured in the process *m* of any shift *j*. According to *Q*_*jm*_ and *G*_*jm*_, Eq (10) calculate the operation time assigned to any employee *P*, which is equal to the sum of the operation time of the working procedure in which the team is located divided by the corresponding number of people. Eq (11) uses the 0–1 variable *Y*_*pjm*_ to indicate whether the employee *P* is configured on the working procedure *M* of the shift *J*. In Eq (12), the decision variable *X*_*ij*_ indicates whether the workpiece *I* is assigned to the shift *J*.

## 3. Model solution based on algorithm

### 3.1 NSGA-II algorithm steps

Genetic algorithm (GA) is a random search algorithm, which draws lessons from natural selection and natural genetic mechanism in biology. Rosenberg mentioned that genetic-based search algorithm can be used to solve multi-objective optimization problems [31]. with the development of multi-objective genetic algorithm, Srinivas and Deb put forward NSGA (non-dominated sorting genetic algorithm) in 1995. It has the advantages of uniform distribution of non-inferior optimal solutions, allowing multiple different equivalent solutions, and is widely used in practical problems. In view of the disadvantages of NSGA, such as high computational complexity, lack of elite decision, and great dependence on shared parameters [32], Deb et al. [33] proposed an improved algorithm NSGA-II. NSGA-II algorithm removes shared parameters and introduces elite decision-making, and the computational complexity is reduced from O(MN3) to O(MN2). The flow chart of NSGA-II algorithm is shown in Fig 1, and the basic steps are as follows:

1. Initialize population *P*_*t*_ (*t* = 0): Use the algorithm to randomly generate a parent population with a population size of *n*.
2. Generation of the first-generation population: Refers to the pareto classification and calculation of individual crowding degree by initializing the population, so as to produce the first-generation population.
3. Binary tournament selection is an elite strategy of NSGA-II algorithm, which can select individuals with excellent genetic characteristics.
4. Fusion of parent *P*_*t*_ and offspring *O*_*t*_: In order to avoid the loss of parent individuals with excellent genetic characteristics in the process of generating offspring, the parent and offspring are fused, and then the excellent individuals of scale *n* are selected from the fused population to continue inheritance.

**Fig 1:** Flowchart of NSGA-II algorithm.

### 3.2 NSGA-II-EDSP algorithm steps

SPT rule (shortest processing time) and EDD rule (earliest due date) are commonly used in job shop scheduling when there is a due date. In this paper, the NSGA-II algorithm is improved by combining SPT and EDD rules. First, the jobs are sorted based on EDD rules, then the jobs are sorted based on SPT rules, and finally the jobs are sorted based on NSGA-II algorithm. The algorithm is named NSGA-II-EDSP (NSGA-II- Earliest due Shortest Processing). The detailed process is as follows:

Step1: An initial population P_0_ with the size of N is randomly generated, and the P 0 is sorted by the EDD algorithm (the shorter the delivery time is, the earlier the delivery time is);
Step 2: according to the sorting result of P_0_, the SPT rule is used to modify the sorting result (the shorter the processing time is, the earlier the processing time is within the current delivery time range), and the adjusted initial chromosome code is obtained;
Step 3: the offspring population Q_0_ was generated by genetic evolution (crossover and mutation), and Q_0_ was regarded as the initial population, so that t = 0; After that, the offspring and parents were merged;
Step 4: calculate the two objective total delay and standard deviation of each solution, and sort *Rt* non dominated to get an ordered solution space, and then Pareto layer all the solutions;
Step 5: select the first n solutions in the ordered solution space in step 4 as the parent of the next generation population *P*_*t*+1_;
Step 6: take tournament selection for *P*_*t*+1_, and carry out genetic evolution operation (crossover and mutation) to produce offspring *Q*_*t*+1_;
Step 7: perform the next generation evolution operation, let *t* = *t*+1. If the maximum number of iterations is reached, the Pareto optimal solution set is output; otherwise, Step 2 is returned to cycle until the end of iteration.

### 3.3 NSGA-II-KES algorithm steps

In the process of solving genetic algorithm, the selection of subpopulation is often random and extremely unstable. According to the research, the initial value of the subpopulation will greatly affect the final solution of the subpopulation, and also affect the convergence rate of the subpopulation, and the degree of individual aggregation in the subpopulation will also affect the probability of obtaining the optimal solution. Considering this feature, this paper first performs the initial K-Means clustering on the population number to get the classified population, and then solves it based on NSGA-II-EDSP algorithm. The algorithm is named NSGA-II-KES (NSGA-II- K Earliest Shortest). The detailed process is as follows:

Step 1: randomly generate an initial population P_0_ with size n, classify P_0_ by K-means clustering, measure the distance by Euclidean distance, and get K populations;
Step 2: rearrange the individuals of K populations to get the initial chromosome population Q_0_;
Step 3: execute NSGA-II-EDSP algorithm flow.

### 3.4 NSGA-II-QKES algorithm steps

Crossover operator is a very important operation in genetic algorithm, which is the main way of population evolution. In the crossover operator, the population crossover rate is the key parameter, and the selection of crossover rate can affect the efficiency and performance of the algorithm to a greater extent. Based on this, reinforcement learning is used to realize the parameter self-learning process of genetic algorithm, which mainly acts on the selection and setting of crossover rate to realize the self-learning of population crossover rate. The algorithm is named NSGA-II-QKES (NSGA-II- Q K Earliest Shortest). The detailed process is as follows:

Step 1: execute Step 1 and Step 2 of NSGA-II-KES algorithm and Step 1 and Step 2 of NSGA-II-EDSP algorithm;
Step 2: the reward and punishment mechanism of reinforcement learning is determined as follows: the best fitness and average fitness become larger, only the best fitness and average fitness become larger, and the optimized crossover rate is obtained;
Step 3: execute Step 4 and Step 7 of NSGA-II-EDSP algorithm.

### 3.5 Chromosome coding rules

In nature, the chromosomes of living things are usually coupled together in pairs. During its evolution, the father and mother each provided half of the chromosomes to form a new genome. In this problem, when the workpiece is assigned to the shift, the processing sequence in the shift should be considered at the same time. The coding form of single gene model can’t express its solution well. Therefore, this paper adopts double chromosome coding method for coding. The first chromosome is coded with its workpiece number (I) as the gene, which controls the processing order of its individual in the evolution process. The sequence before and after the workpiece number indicates its processing order priority. The second chromosome is coded with the shift number (*j*) as the gene, indicating the operation result of its grouping, as shown in Table 1.

**Table 1:** Double chromosome coding.

Job order	5	13	…	16	3	…	4	19	…	9	21
Grouping results	3	1	…	4	2	…	1	2	…	4	3

### 3.6 Calculation of crowding degree

For the population with the size of *P*, all individuals of the population can be layered by the non-dominated sorting algorithm, and several layers of non-dominated solution sets (Pareto Front) can be obtained. Crowding degree in niche technology is used to maintain diversity of population distribution. The congestion degree of each solution can be expressed by the distance between two adjacent solutions on the corresponding non-dominated solution set on each target. Because the measurement units of different targets are different, the normalized method is used to map the data to the range of 0~1. In this paper, the congestion degree of the solution obtained by the algorithm is calculated as follows:

Let *γ f* is the non-dominated solution set of level *f* obtained by the algorithm, *X*_*i*_ is the solution in *γ f*, let *n* is the number of solutions in *γ f*, *C*_*i*_ and *B*_*i*_ are the delay coefficient and equalization coefficient after normalization of solution *X*_*i*_, and *L*_*i*_ is the congestion degree of *X*_*i*_.


$$L_{i}=\{\begin{array}{l} \;2\sqrt{2},\;(N=1)\\ \;\sqrt{{\left(C_{i}-C_{i+1}\right)}^{2}+{\left(B_{i}-B_{i+1}\right)}^{2}},\;(N\geq 2,\;i=1)\\ \;\sqrt{{\left(C_{i-1}-C_{i}\right)}^{2}+{\left(B_{i-1}-B_{i}\right)}^{2}},(N\geq 2,\;i=N)\\ \sqrt{{\left(C_{i-1}-C_{i+1}\right)}^{2}+{\left(B_{i-1}-B_{i+1}\right)}^{2}},(N\geq 2,\;1<i<N) \end{array}$$ (13)

The formula for calculating the congestion degree *L*_*i*_ is given in Eq (13). When *N* = 1, that is, *γ f* has only one solution, then its congestion degree is $2\sqrt{2}$. When *n* is greater than 2, that is, when *γ f* has multiple solutions, the congestion degree of the first and last solutions is taken as the normalized distance between one of its adjacent solutions, and the congestion degree of other solutions is taken as the normalized distance between the two solutions before and after it.

### 3.7 Evolutionary operation

After all the solutions are sorted by non-domination, the level *f* of non-domination solution set and its crowding degree *L*_*i*_ of solution *X*_*i*_ can be obtained. They are sorted according to the following partial ordering relationship, and the crowding distance in niche technology is used to maintain the diversity of population distribution. Adopt binary tournament and elite retention strategy to select individuals for evolutionary operation. The PMX method was used to perform the same crossover operation on the two chromosomes. In the process of mutation, the first chromosome is exchanged in position to ensure the non-repetition and loss of the workpiece, and the second chromosome is mutated at a single point, and its processing team is re-selected.

## 4. Example verification

### 4.1 Example design

In order to verify the effectiveness of the proposed model and algorithm, an example is designed. Table 2 shows the weekly orders and the processing time and delivery rules of their workpieces, and Table 3 shows the current distribution of team members.

**Table 2:** Rules of weekly order table.

Factor	Classification and value taking
Delivery date of a single workpiece	Rand(1,2)* sum of workload of single product
Number of artifacts in weekly orders	U(100, 150)
Process 1: component installation (hours)	U(25, 35)
Operation 2: primary wiring (hours)	U(30, 45)
Step 3: Secondary wiring (hours)	U(30, 45)
Process 4: copper bar installation (hours)	U(30, 40)

**Table 3:** Distribution of team members.

Team name/person	Component installer	Primary wiring personnel	Secondary wiring personnel	Copper bar installer
Team 1	7	6	9	6
Team 2	8	7	9	5
Team 3	9	5	8	8
Team 4	8	7	6	7

According to the rule of weekly orders in Table 2, the orders with 100,110,120 and 150 workpieces were generated respectively, which were solved by the algorithm combined with the distribution of team members in Table 3.

### 4.2 Model application and solution

Through the pre-experiment, the population size of the parameters is set to 100, the number of iterations is 150, the crossover rate is 0.9, and the variation rate is 0.1, which can achieve a better solution effect. The algorithm is implemented in C# language, the running environment is Intel (R) Core (TM) i7-9750HQ CPU @ 2.60GHz, and the running memory is 12GB. Fig 2 shows the solution results of orders with 100, 110, 120 and 150 workpieces and their Pareto front. Each point in the graph represents a solution, that is, a scheduling scheme. At the same time, Table 4 gives the details of the final Pareto frontier solutions of four examples, and the workpiece allocation of the solution (T = 33.20, σ = 15.8) in the order of 110 workpieces was shown in Table 5.

**Fig 2:** Pareto diagram after solving each imitation case.

**Table 4:** Pareto frontier data table after solving each imitation case.

100 pieces Pareto frontier solution		110 pieces Pareto frontier solution		120 pieces Pareto frontier solution		150 pieces Pareto frontier solution	
T	σ	T	σ	T	σ	T	σ
4.11	11.53	70.21	13.40	140.34	23.02	175.43	28.77
15.41	10.31	79.88	11.97	528.57	12.48	660.71	15.60
5.23	10.39	106.56	11.42	281.88	13.15	352.35	16.44
0.00	12.55	106.42	11.68	81.04	23.49	101.30	29.36
0.48	11.70	37.12	14.74	219.48	14.49	274.35	18.11
		33.20	15.80	140.35	18.46	175.44	23.07
		131.15	10.51	162.20	14.93	202.75	18.66
		0.00	46.55	464.74	12.83	580.92	16.03
						654.81	16.03
						340.39	16.91

**Table 5:** Two chromosomes of solution (T = 33.20, σ = 15.8) in order with 110 workpieces.

1	65	52	107		23	109	47	21	103	110	11	33	99	83	97	79	73	84	92	49	6	88	45	82	54	101	17	40	85	98
			100		96	31	104	18	81	75	95	50	46	86	70	61	55	105	30	5	42	19	58	69	90	94	89	108	56	22
			35		53	63	62	2	28	77	72	57	80	44	43	51	102	59	87	67	48	9	25	91	37	32	60	15	29	36
			71		26	38	24	68	34	20	16	8	12	13	93	66	4	41	7	39	10	74	1	64	106	78	76	3	14	27
2	4	3	4		3	1	3	4	3	3	2	1	4	4	4	2	1	3	2	4	1	1	4	2	3	1	1	2	4	1
			3		2	4	1	2	2	1	4	2	4	1	3	4	3	4	1	4	4	1	4	3	4	4	2	4	1	1
			2		2	2	1	2	1	3	1	4	1	4	2	3	1	1	2	2	4	3	1	1	2	3	2	2	1	4
			2		3	3	3	1	2	2	4	3	1	4	3	3	1	3	4	4	1	2	3	3	3	3	2	3	2	4
Order assigned by team 1				109 >> 33 >> 73 >> 6 >> 88 >> 101 >> 17 >> 98 >> 104 >> 75 >> 86 >> 30 >> 19 >> 56 >> 22 >> 62																										
				>> 28 >> 72 >> 80 >> 102 >> 59 >> 25 >> 91 >> 29 >> 68 >> 12 >> 4 >> 10 >>																										
Order assigned by team 2				11 >> 79 >> 92 >> 82 >> 40 >> 96 >> 18 >> 81 >> 50 >> 89 >> 35 >> 53 >> 63 >> 2 >> 43 >> 87 >> 67																										
				>> 37 >> 60 >> 15 >> 71 >> 34 >> 20 >> 74 >> 76 >> 14 >>																										
Order assigned by team 3				52 >> 23 >> 47 >> 103 >> 110 >> 84 >> 54 >> 100 >> 70 >> 55 >> 69 >> 77 >> 51 >> 9 >> 32 >> 26																										
				>> 38 >> 24 >> 8 >> 93 >> 66 >> 41 >> 1 >> 64 >> 106 >> 78 >> 3 >>																										
Order assigned by team 4				65 >> 107 >> 21 >> 99 >> 83 >> 97 >> 49 >> 45 >> 85 >> 31 >> 95 >> 46 >> 61 >> 105 >> 5 >> 42 >>																										
				58 >> 90 >> 94 >> 108 >> 57 >> 44 >> 48 >> 36 >> 16 >> 13 >> 7 >> 39 >> 27 >>																										

### 4.3 Result analysis

It can be seen from Fig 2 that with the increase of the number of workpieces, the points (solutions) constituting the Pareto front also increase, and the Pareto front range becomes wider and wider. The reason is that when the total processing time required by an order is less than the total processing capacity of its workshop, there may be a solution of total delay time *T* = 0. These solutions will be dominated by one of them, and with the smaller number of workpieces (total processing time). The larger the number it dominates, as shown in Fig 2*A*–2*D*. When the total processing time of the workpiece is greater than the total processing capacity of the workshop, there will be no solution with *T* = 0, and the solution obtained by the algorithm will be more fully extended in two dimensions, so the Pareto front will be wider.

According to the solution results of each imitation in Table 4, when the total processing time of the workpiece meets the processing capacity of the total workshop, there may be a solution of *T* = 0, but it is difficult to find a solution that makes the workload difference between employees 0 (i.e., *σ* = 0). At this time, because of the fixed operation mode and quality tracking system of the production line, the workload of employees cannot be further distributed.

### 4.4 Algorithm comparison

The comparison of two heuristic operator algorithms is introduced in this section. For the performance evaluation of multi-objective algorithm, the number and quality of solutions at Pareto front level obtained by the algorithm are mainly considered. In this paper, order of magnitude index, span index and error ratio index are used to analyze and compare.

Table 6 lists the number of non-dominant solutions on Pareto front obtained by the three algorithms on different types of imitations. Among them, the category of the example is listed in the type column. For example, *J*_1_*F*_1_ indicates the working environment in which the number of workpieces *J*_1_ = 110 and the personnel distribution form is *F*_1_. Fig 3 shows the trend of the maximum number of solutions for different cases. From the perspective of J1, J2 and J3, we can see that with the increase of the number of workpieces, the number of solutions for each algorithm increases. Because with the increase of the number of jobs, the delay time index of the obtained solution will expand, and more disposable solutions will appear. From the perspective of F1, F2, F3 distribution, the difference of the overall distribution is small, only the number of average solutions of F1 is relatively small. NSGA-II-EDSP, NSGA-II-KES, and NSGA-II-QKES have excellent performance in finding solutions, which are improved by 18.27%, 22.0% and 22.26% respectively.

**Fig 3:** Algorithm comparison chart.

**Table 6:** Comparison of the number of non-dominant solutions obtained by each algorithm.

Type	NSGA-II	NSGA-II-EDSP	NSGA-II-KES	NSGA-II-QKES
J1F1	7.86	8.68	9.68	9.72
J1F2	8.86	11.26	10.68	10.69
J1F3	8.43	10.76	11.21	11.53
J2F1	10.86	13.68	13.40	13.40
J2F2	13.00	16.82	16.96	16.97
J2F3	14.00	18.25	19.82	19.91
J3F1	17.57	21.39	22.25	22.28
J3F2	13.71	15.03	15.09	15.21
J3F3	16.71	19.81	19.81	19.83

The span values of each algorithm in different types of imitation cases are shown in Table 7. Fig 4 shows the maximum span variation of each algorithm for different cases. When the number of workpieces exceeds the total processing capacity of the factory, some orders will not be completed in time, resulting in delay. The more the number of workpieces exceeds the total processing capacity, the more serious the delay. From the perspective of types J1, J2 and J3, it can be seen that with the increase of the number of workpieces, the Pareto frontier span of each algorithm is gradually increasing, and the overall performance preference of NSGA-II-EDSP, NSGA-II-KES, and NSGA-II-QKES algorithms. As can be seen directly from Fig 4, NSGA-II-EDSP, NSGA-II-KES, and NSGA-II-QKES show good range search ability, and their search ability is relatively stable, with an average improvement of 13.07%, 15.22% and 17.55% respectively.

**Fig 4:** Algorithm comparison chart.

**Table 7:** Comparison of span values of various algorithms.

Type	NSGA-II	NSGA-II-EDSP	NSGA-II-KES	NSGA-II-QKES
J1F1	1.09	1.25	1.27	1.32
J1F2	1.10	1.32	1.35	1.36
J1F3	1.11	1.27	1.30	1.34
J2F1	1.14	1.19	1.21	1.22
J2F2	1.26	1.49	1.52	1.56
J2F3	1.24	1.51	1.54	1.57
J3F1	1.29	1.45	1.48	1.49
J3F2	1.26	1.40	1.38	1.41
J3F3	1.26	1.39	1.41	1.43

The quality of the solution is one of the main indexes to evaluate the performance of the algorithm. In this paper, the error ratio index (ER) is used to express the difference between the solution and the real Pareto front. When ER is between [0,1], the smaller the error is, the smaller the distance between ER and the real front solution is, the better the solution is. According to the data in Table 8, the minimum Er value of NSGA-II is 0.30, while the minimum ER values of NSGA-II-EDSP, NSGA-II-KES, and NSGA-II-QKES are only 0.26, 0.24 and 0.23. It shows that NSGA-II-QKES algorithm is relatively stable when the algorithms are in the worst condition. The maximum Er value of each algorithm is shown in Fig 5. It can be clearly seen from the figure that the improved algorithm has absolute advantages and stability in solving quality. The average effect of NSGA-II-EDSP, NSGA-II-KES, and NSGA-II-QKES were increased by 14.56%, 15.16% and 15.67% respectively.

**Fig 5:** Algorithm comparison chart.

**Table 8:** Comparison of error ratio of each algorithm.

Type	NSGA-II	NSGA-II-EDSP	NSGA-II-KES	NSGA-II-QKES
J1F1	0.74	0.63	0.64	0.64
J1F2	0.57	0.48	0.47	0.46
J1F3	0.52	0.47	0.46	0.46
J2F1	0.30	0.26	0.24	0.23
J2F2	0.52	0.46	0.47	0.47
J2F3	0.57	0.49	0.48	0.48
J3F1	0.61	0.51	0.51	0.51
J3F2	0.71	0.59	0.60	0.59
J3F3	0.46	0.39	0.38	0.38

## 5. Conclusion

In this paper, according to the characteristics of parallel flow shop scheduling, considering the influence of scheduling scheme on the workload imbalance of operators, a method of describing the employee’s work balance degree by work standard deviation is proposed, and a multi-objective scheduling optimization model of parallel flow shop is established. Based on the improved NSGA-II algorithm, the model is solved, and its chromosome coding mode, the calculation of congestion degree gives detailed solving steps. The multi-objective scheduling optimization model proposed in this paper and an example of solving algorithm design are used for simulation research. The results show that the algorithm proposed in this paper has achieved better optimization results in order delivery and employee assignment, and compared with the previous random assignment method. It has more rationality and practical guiding significance. The follow-up study can further consider the psychological impact of scheduling changes on employees, so as to improve their work enthusiasm.

## Supporting information

S1 Data (XLSX)
